The article "Combined Therapy with Traditional Chinese Medicine and Antiplatelet Drugs for Ischemic Heart Disease: Mechanism, Efficacy, and Safety" was published in 2021. Journal: Evid Based Complement Alternat Med.

# Combined Therapy with Traditional Chinese Medicine and Antiplatelet Drugs for Ischemic Heart Disease: Mechanism, Efficacy, and Safety

**DOI:** 10.1155/2021/9956248

**Published:** 2021-10-27

**Authors:** Zongliang Yu, Xiaoya Li, Xiaonan Zhang, Dan Li, Yimeng Gu, Min Wu, Longtao Liu

**Affiliations:** ^1^Xiyuan Hospital, China Academy of Chinese Medical Sciences, Beijing, China; ^2^National Clinical Research Center for Chinese Medicine Cardiology, Xiyuan Hospital, China Academy of Chinese Medical Sciences, Beijing, China; ^3^Graduate School of Beijing University of Chinese Medicine, Beijing, China; ^4^Guang'an Men Hospital, China Academy of Chinese Medical Sciences, Beijing, China

## Abstract

Ischemic heart disease is a significant risk factor that threatens human health, and antiplatelet drugs are routinely used to treat cases in clinical settings. Chinese medicine for promoting blood circulation and removing blood stasis (PBCRBSCM) can often be combined with antiplatelet drugs to treat ischemic heart disease. PBCRBSCM can inhibit platelet adhesion, activation, and aggregation; moreover, PBCRBSCM in combination with antiplatelet drugs exerts antiplatelet effects. The mechanism is related to several factors, including the inhibition of platelet activation and aggregation, improvement of the hemodynamic status and coagulation function, and correction of metabolism and inflammation. PBCRBSCM can also regulate the absorption and metabolism of conventional antiplatelet drugs and protect the gastric mucosal epithelial cells against damage induced by conventional antiplatelet drugs. Randomized controlled trials have confirmed that PBCRBSCM preparations and the active ingredients in these preparations can reduce resistance to aspirin and clopidogrel so that the combination of these drugs can exert their antiplatelet effects. In the perioperative treatment of patients with stable angina pectoris, unstable angina pectoris, and acute coronary syndrome undergoing percutaneous coronary intervention therapy, preparations of the active ingredients of PBCRBSCM combined with antiplatelet drugs and other conventional Western medicine treatments have been proven effective. The efficacy and safety of such combinations have also been extensively verified. Considerable progress has been made to understand the antiplatelet mechanism of PBCRBSCM. However, most clinical studies had problems, such as limited sample size and inappropriate research design, which has limited the translational use of PBCRBSCM in antiplatelet therapy. A large-scale, multicenter, randomized controlled study with cardiovascular events as the endpoint is still to be conducted to provide evidence for the combined application of PBCRBSCM and antiplatelet drugs in the prevention and treatment of ischemic heart disease.

## 1. Introduction

Ischemic heart disease is an important risk factor that endangers human health. The rupture of vulnerable plaques and secondary thrombosis are the main causes of acute cardiovascular events [1–3]. Adhesion, activation, and aggregation of platelets are important in regulating cardiovascular processes [4, 5]. Clinically, the use of antiplatelet drugs has become an important means for the prevention and treatment of cardiovascular diseases. However, with the extension of the application time and the combination of multiple drugs, the effectiveness and safety of antiplatelet drugs have attracted clinical attention [6–8]. Recent studies have found that Chinese medicine has a good antiplatelet effect and can be used in combination with conventional antiplatelet drugs to reduce the occurrence of adverse drug reactions [9]. Research on PBCRBSCM is one of the most active fields of investigation that deals with ischemic heart disease and the treatment using integrated traditional Chinese and Western medicine [10]. However, there is a paucity of systematic reviews delineating the antiplatelet mechanism of PBCRBSCM and the role of combination drugs in ischemic heart disease. In this article, we present a detailed study on the efficacy and safety of PBCRBSCM in combination with conventional antiplatelet agents to treat ischemic heart disease.

## 2. The Mechanisms Underlying the Antiplatelet Effect of PBCRBSCM

### 2.1. Inhibiting Platelet Adhesion

Platelet adhesion is the initial stage of thrombosis [11]. Studies have shown that a variety of PBCRBSCMs and their components can play an important role in platelet adhesion. Tian et al. confirmed that, in rats, baicalein could inhibit platelet adhesion induced by a variety of G protein-coupled receptor agonists [12]. Kasimu et al. found that the ethyl acetate extract of *Salvia miltiorrhiza* root inhibits adenosine diphosphate- (ADP-) induced rabbit platelet adhesion and that the mechanism involves the downregulation of von Willebrand factor (vWF) expression [13]. Studies on Danhong and Xuebijing injections have also confirmed that PBCRBSCM inhibits platelet adhesion by downregulating the expression of vWF [14, 15]. Another study found that salvianolic acid B inhibits the binding of integrin *α*2*β*1 to platelets and thereby prevents the interaction of soluble integrin *α*2*β*1 with immobilized collagen in a solid-phase binding assay [16, 17].

Protecting the functional integrity of the vascular endothelium is important for antiplatelet adhesion. Studies have shown that *Panax notoginseng* saponins reduce advanced glycosylation end product-induced apoptosis of human umbilical vein endothelial cells (HUVECs) by upregulating silent mating type information regulation 2 homolog 1 (SIRT1) [18]; these saponins also protect the microvessels of the brain by activating the phosphoinositide 3-kinase (PI3K)/Akt/nuclear factor erythroid 2-related factor 2 (Nrf2) antioxidant signaling pathways [19]. Studies on paeoniflorin have also confirmed its vasoprotective effects [20, 21]. Ligustrazine has an inhibitory effect on platelet adhesion, and its mechanism involves the inhibition of p38 mitogen-activated protein kinase (MAPK) and nuclear factor-kappa B (NF-*κ*B) signaling pathways to downregulate endothelial inflammation [22]. Other studies have revealed that peach kernels and safflower extracts regulate the production of nitric oxide (NO) in endothelial cells, thereby inhibiting platelet adhesion and aggregation [23, 24]. Therefore, PBCRBSCMs and their active ingredients have a definite antiplatelet effect. The mechanism mainly involves the downregulation of vWF, interference with collagen receptors, and protection of the vascular endothelium. PBCRBSCMs and their active ingredients with antiplatelet effects are shown in Figures 1 and 2.

### 2.2. Inhibiting the Activation and Degranulation of Platelets

ADP binds to the G protein-coupled receptors P2Y purinoceptor 1 (P2Y1) and P2Y purinoceptor 12 (P2Y12) localized on the platelet surface, causing platelet activation and further release of ADP. P2Y1 activates phospholipase C*β*, leading to an increase in intracellular Ca2+ levels. P2Y12 activation reduces the level of cyclic adenosine monophosphate (cAMP), leading to the recruitment of additional platelets at the injured site [25].

Many studies have confirmed that PBCRBSCM exerts antiplatelet effects by inhibiting the ADP pathway. Huang et al., using a mouse arterial thrombosis model, observed that salvianolic acid A prolonged the time of mesenteric artery occlusion in wild-type mice. Further studies found that salvianolic acid A inhibited ADP-induced platelet activation by inhibiting platelet spreading on the fibrinogen (FIB) matrix. This mechanism may be related to the regulation of PI3K and Akt phosphorylation [26]. Serum studies of patients with type 2 diabetes also confirmed that salvianolic acid A reduces the expression of procaspase-activating compound-1 (PAC-1) and P-selectin (CD62P) and inhibits platelet activation [27]. Studies have shown that tanshinone IIA selectively inhibits ADP-induced platelet activation and aggregation in rats. Further experiments on the collected platelet lysate showed that tanshinone IIA primarily exerts its antiplatelet effect by regulating tubulin acetylation and inhibiting extracellular signal-regulated kinase- (Erk-) 2 phosphorylation [28]. A docking study showed that cryptotanshinone and tanshinone IIA are Gi-coupled P2Y12 receptor antagonists. This attribute of receptor antagonism may be the key mechanism by which cryptotanshinone and tanshinone IIA inhibit platelet activation in rats [29]. Studies on the inhibition of platelet activation and aggregation by notoginsenoside Ft1 also confirmed that it binds to P2Y12 receptors and increases the phosphorylation of PI3K and Akt downstream of the P2Y12 channel. Some active ingredients widely present in a variety of traditional Chinese medicines may also inhibit platelet activation by inhibiting the ADP pathway. For example, studies on apigenin have confirmed its ability to resist platelet aggregation induced by arachidonic acid (AA) and ADP [30]. Moreover, quercetin and resveratrol inhibit thrombin-induced platelet ADP and adenosine triphosphate (ATP) secretion in a concentration-dependent manner [31].

Following platelet activation, the activated phospholipase A2 cleaves membrane phospholipids and frees AA, which is then converted to prostaglandin G2 and H2 (PGG2 and PGH2) by the action of cyclooxygenase (COX). The active ingredients of several PBCRBSCMs can exert antiplatelet activation effects by inhibiting the AA pathway. Cheng et al. constructed a rat middle cerebral artery occlusion model and showed that the active compound in Dan Zhi tablets reduced the infarct size and neurological score of rats and inhibited AA-induced platelet aggregation [32]. Similarly, hirudin effectively inhibited AA-induced platelet activation and aggregation [33]. Thromboxane B2 (TXB2) and 6-keto-prostaglandin F1 alpha (PGF1*α*) are stable metabolites of TXA2 and prostaglandin I2 (PGI2), respectively. A study found that notoginsenoside Fc inhibited the thrombin-induced synthesis of diacylglycerol-protein kinase C- (PKC-) thromboxane A2 (TXA2) and inositol 1,4,5-trisphosphate and downregulated the expression of TXB2 [34]. Dang et al. established a rat model of acute blood stasis to verify the antiplatelet activity of Sheng-Nao-Kang decoction (RSNK); they confirmed that treatment with RSNK significantly inhibited the level of TXB2 in the blood stasis model rats and upregulated the level of 6-keto-PGF1*α*, which inhibited platelet activation and aggregation [35]. Zhang et al. synthesized a paeonol-ozagrel conjugate and verified that its antiplatelet activation effect in a rat model of middle cerebral artery occlusion is related to the inhibition of endothelial inflammation and reduction of TXA2 levels [36]. Experimental studies on ADP-induced platelet aggregation in rabbits and FeCl3-induced common carotid artery thrombosis in rats have revealed that the antiplatelet activation effect of the ethyl acetate extract of Danshen root is related to the reduction of 6-keto-PGF1*α* [13].

In addition, studies have found that ginkgo diterpene lactones inhibit platelet activation and aggregation induced by platelet-activating factor (PAF) and protect the ischemic tissue by downregulating the Toll-like receptor (TLR) 4/NF-*κ*B signaling pathway [37]. Studies with tanshinone IIA sodium sulfonate have also confirmed its role in platelet aggregation induced by PAF [38]. Studies using curcumadione extracts obtained from turmeric also confirmed its inhibitory effect on PAF-induced platelet activation and aggregation [39]. In general, PBCRBSCM inhibits platelet activation mainly by blocking the ADP, P2Y1, and P2Y12 receptors on platelets and inhibiting the synthesis of PAF and TXA2, thereby improving the microcirculation of blood and inhibiting the degranulation of platelets secretion.

### 2.3. Inhibiting Platelet Aggregation

cAMP and cyclic guanosine monophosphate (cGMP) inhibit platelet aggregation induced by increased Ca2+ levels [40, 41]. The increase in intracellular Ca2+ and the decrease in cAMP caused the activation of glycoprotein IIb/IIIa (GP IIb/IIIa), which makes it receptive to binding by FIB and vWF, eventually resulting in thrombosis [42]. Therefore, inhibiting the increase in intracellular Ca2+ as well as increasing the level of cAMP/cGMP is an important way to prevent platelet aggregation.

Previous studies have found that cordycepin inhibits collagen-induced platelet aggregation and inhibits the increase in Ca2+ levels and the production of TXA2. Some studies have also found that cordycepin increases the levels of cAMP and cGMP in collagen-stimulated platelets. Therefore, the inhibitory effect of cordycepin on platelet aggregation may be related to the downregulation of Ca2+ and increase in cAMP/cGMP production [43]. Studies on curcumone, curcumol, and other traditional Chinese medicine extracts of *Curcuma* have also confirmed that these *Curcuma* compounds inhibit the mobilization of Ca2+ and regulate the expression of cAMP, thereby exerting an antiplatelet aggregation effect [39, 44]. In the arteriovenous shunt model, salvianolic acid A significantly inhibited the activation and aggregation of platelets stimulated by various agonists, and its underlying mechanism may involve the induction of cAMP [45]. Similarly, dimethyl fumarate, resveratrol, and curcumin have been shown to regulate cAMP levels [46, 47].

The GP IIb/IIIa receptor (integrin-*α*IIb/*β*3) is an integrin protein localized on the surface of platelets. FIB is the main ligand of the GP IIb/IIIa receptor. Under the action of thrombin, FIB is converted into fibrin, which crosslinks adjacent platelets to form a stable platelet aggregate, which is the final stage of thrombosis [48]. Studies have revealed that quercetin is widely present in various PBCRBSCMs. It can inhibit the activation of integrin-*α* IIb/*β*3 and promote the production of cAMP and vasodilator-stimulated phosphoprotein. This mechanism involves the inhibition of MAPK phosphorylation [49]. The extraction and pharmacological studies of the active ingredients of the traditional Chinese medicine red peony root also confirmed the regulation of FIB in platelet aggregation inhibition, as well as the inhibitory effect of paeoniflorin on platelet aggregation [50]. In addition to FIB, vWF can also bind to GPIIb/IIIa to crosslink adjacent platelets. Yin et al. used phenylhydrazine-induced thrombosis to construct a zebrafish thrombosis model and explored the antiplatelet aggregation activity of *Salvia miltiorrhiza* and *Panax notoginseng*. Their results confirmed that rosmarinic acid, shikimic acid, and salvianolic acid B present in these extracts showed good antiplatelet aggregation effects. This mechanism of inhibiting platelet aggregation involves the downregulation of PKC and vWF expression [51]. Overall, the antiplatelet aggregation effect of PBCRBSCM is definite, and its mechanism mainly involves inhibiting the levels of Ca2+/increasing the levels of cAMP, inhibiting the activation of integrin-*α* IIb/*β*3, and downregulating the expressions of FIB and vWF. The mechanisms underlying the antiplatelet effects of PBCRBSCM are presented in Figure 3.

## 3. The Mechanisms Underlying the Combined Application of PBCRBSCM and Antiplatelet Drugs

### 3.1. Combination Medication Exerts Antiplatelet Effect

Recent studies have shown that PBCRBSCM can be combined with conventional drugs, such as aspirin and clopidogrel, to exert antiplatelet effects [52, 53].

A study confirmed that the antiembolism effect of Taoren Chengqi decoction is related to the concentration-dependent inhibition of platelet activation [54]. Similarly, Hsu et al. confirmed the protective effect of Taoren Chengqi decoction alone or in combination with aspirin on cerebral infarction. Their study revealed that the expression levels of tumor necrosis factor-alpha (TNF-*α*) and c-Jun N-terminal kinase in the ischemic area of rats treated with Taoren Chengqi decoction alone or in combination with aspirin were significantly reduced and that the expression of caspase-3 and Bcl2-associated X protein (Bax) was downregulated [55]. Wang et al. explored the effects of leech extract on hemorheology and metabolic disorders in rats through automatic hemorheology analysis and liquid chromatography-mass spectrometry (LC-MS) nontargeted metabolomics assays. The results showed that a medium dose (2.5 g/kg) of leech extract had the same effect on hemorheology and histopathological parameters of rats as aspirin and that the leech extract could significantly improve the metabolic disorders related to high blood viscosity [56]. Similarly, the active ingredients of traditional Chinese medicines, such as Moutan bark, peach kernel, and safflower, can inhibit platelet aggregation when combined with aspirin [57, 58]. Other studies found that Angelica and safflower have antithrombotic effects on venous thrombosis and pulmonary embolism, but that they could not significantly enhance the antithrombotic effects of clopidogrel in cases of arterial thrombosis and pulmonary embolism [59]. Several experimental studies have confirmed that the mechanism of action of some PBCRBSCMs and their active ingredients when combined with conventional antiplatelet drugs is mainly related to inhibition of platelet activation and aggregation, improvement of hemodynamic status, and correction of metabolism and inflammation.

### 3.2. Regulating the Metabolism of Antiplatelet Drugs

Some PBCRBSCMs have been found to modulate the pharmacokinetic parameters of antiplatelet drugs and jointly exert antiplatelet effects [60, 61].

Xiao et al. used LC-MS/MS to explore the effects of Danshen, *Pueraria lobata*, Angelica, and Chuanxiong on the serum metabolites of aspirin and clopidogrel—dual antiplatelet drugs. The results showed that the coadministration of *Pueraria lobata* and Angelica changed the pharmacokinetics of aspirin and clopidogrel and increased the concentration of aspirin and clopidogrel in the blood. Furthermore, *Salvia miltiorrhiza*, *Pueraria lobata* root, and Angelica gavage showed a significant inhibitory effect on rCyp2c11 and carboxylesterase activity but without any significant effect on aspirin esterase activity [62]. Tian et al. determined the concentration of salicylic acid in the blood after aspirin was administered in combination with notoginseng leaf glycosides. The results showed that notoginseng leaf glycosides increased the concentration of salicylic acid in the blood. Further, in vitro transporter assays using a monolayer of Madin-Darby canine kidney cells showed that notoginseng leaf glycosides in combination with aspirin significantly increased the apparent permeability coefficient, confirming that notoginseng leaf glycosides promoted the absorption of aspirin from the gastrointestinal tract [63]. Interestingly, another rat study found that the combination of notoginsenoside and aspirin increased the concentration of notoginseng saponins and ginsenosides in the blood. The mechanism involves aspirin-mediated destruction of tight junction proteins, with consequent widening of intercellular spaces, which subsequently increases the absorption of *Panax notoginseng* saponins [64]. Thus, PBCRBSCM can jointly exert antiplatelet effects by modulating the pharmacokinetic parameters of conventional antiplatelet drugs, while antiplatelet drugs can also affect the absorption and metabolism of PBCRBSCMs.

### 3.3. Reducing Gastric Mucosal Damage

Antiplatelets increase the risk of gastrointestinal bleeding, and their mechanism involves the reduction of COX activity, endogenous prostaglandin synthesis, release of inflammatory factors, and increased gastric mucosal barrier damage.

Studies have found that some PBCRBSCMs and their active ingredients protect the gastric mucosa. Xie et al. found through in vivo studies that traditional Chinese medicine preparations dose-dependently reduced the ulcer focus index in an ethanol-induced rat ulcer model [65]. Wang et al. found that *Panax notoginseng* saponins effectively reduced the damage of human gastric mucosal epithelial cells induced by double antiplatelets and upregulated the expression of prostaglandin E2 (PGE2) and other biological factors. The mechanism is related to the regulation of the PI3K/Akt/vascular endothelial growth factor- (VEGF-) glycogen synthase kinase- (GSK-) 3*β* and ras homolog gene family member A (RhoA) network pathway to reduce the inhibitory effect of dual antiplatelet drugs on the COX/prostaglandin (PG) pathway [66]. Similarly, a study on a rat model of myocardial infarction also confirmed the protective effect of *Panax notoginseng* saponins on aspirin-induced gastric mucosal damage. It is believed that its mechanism of action is related to the increase in 6-keto-PGF1*α* and PGE2 in response to the AA/PG pathway [67]. Li et al. confirmed that Danhong injections reduced aspirin-induced gastric mucosal damage, improved gastric mucus secretion, reduced pepsin activity, and maintained the integrity of the gastric mucosal barrier. In addition, Danhong injection reduced the level of reactive oxygen species in the gastric mucosa and increased the activity of catalase and superoxide dismutase (SOD) [68].

Clinical studies have also confirmed the protective effect of PBCRBSCM against platelet drug-induced gastric mucosal damage. The results of a randomized controlled trial involving 42 patients showed that the dyspepsia symptoms of patients in the *Panax notoginseng* saponins combined with the aspirin group were significantly less than those in the aspirin group alone. Further studies confirmed the inhibitory effect of *Panax notoginseng* saponins on the activity of platelet COX-1 and the downregulation of TXB2, PGD2, and PGE2 expressions [67]. A randomized controlled study of 117 patients with gastrointestinal bleeding after percutaneous coronary intervention has also shown that the protective effect of traditional Chinese medicines on the gastric mucosa is equivalent to that of pantoprazole sodium enteric-coated capsules [69]. Overall, PBCRBSCMs can regulate inflammation pathways and AA/COX/PG pathways, exert a protective effect on gastric mucosal epithelial cells, inhibit the occurrence of ulcers, and reduce gastric mucosal damage induced by conventional antiplatelet drugs.

### 3.4. Protecting the Vascular Endothelium

Endothelial injury is the initiates of platelet adhesion. Studies have found that aspirin reduces oxidative stress damage and the inflammatory response of HUVECs induced by oxidized low-density lipoprotein [70]. Some PBCRBSCMs exert a synergistic effect by protecting the vascular endothelium and regulating the antiplatelet drugs.

Wang et al. constructed an oxidation low-density lipoprotein- (ox-LDL-) induced HUVEC injury model and found that the combination of Panax ginsenoside and dual antiplatelet drugs reduced HUVEC apoptosis and improved the adhesion of platelets to damaged HUVECs. Simultaneously, it increased the concentration of 6-keto-PGF1*α* in the supernatant and the phosphorylation level of Akt protein, which was more effective than dual antiplatelet drugs alone. This suggests that the protective effect of Panax ginsenoside and dual antiplatelet drugs on platelet adhesion may be related to the PI3K/Akt and COX pathways in HUVECs and platelets [71]. Similarly, a study of *Panax notoginseng* saponins combined with double antiplatelets also showed the inhibition of ox-LDL-induced apoptosis of HUVECs and the improvement of platelet adhesion. This mechanism is related to the downregulation of the PI3K/Akt signaling pathway [72]. The mechanisms of the combined application of PBCRBSCM and antiplatelet drugs are shown in Figure 4.

## 4. The Mechanisms of PBCRBSCM Combined with Antiplatelet Drugs in Ischemic Heart Disease

Platelet adhesion, activation, and aggregation are important steps in the formation of intra-arterial thrombosis. Numerous in vivo and in vitro experimental studies have confirmed the antiplatelet activity of PBCRBSCMs and their interaction with antiplatelet drugs. PBCRBSCMs and their active ingredients and antiplatelet drugs are widely used in the clinical treatment of coronary heart diseases [73, 74]. A study comprising 16,856 patients in 37 first-class tertiary hospitals in China showed that the frequency of combined use of Suxiao Jiuxin Pill and aspirin was as high as 50.77%. This shows the degree of combined application of PBCRBSCMs and antiplatelet drugs in ischemic heart disease [75]. Gas chromatography/mass spectrometry (GC-MS) and LC-MS nontargeted metabolic assays confirmed that the combination of Danshen dripping pills and clopidogrel improved the antiplatelet efficacy of patients with coronary heart disease by regulating the metabolites [76]. Another small randomized controlled trial involving 18 patients with coronary heart disease showed that the combined use of *Salvia miltiorrhiza* polyphenolate enhanced the antiplatelet activity of aspirin. Compared with aspirin alone, the combined use of salicylic acid shortened the absorption time of salicylic acid, prolonged the elimination time of salicylic acid, and downregulated the expression of MAPK8, CD62p, and P2Y12 [77]. Generally, clinical research on the antiplatelet mechanism of PBCRBSCMs and their active ingredients combined with conventional drugs needs to be further improved.

Studies have found that antiplatelet drug resistance is a risk factor for cardiovascular events in patients with cardiovascular disease [78, 79]. Reducing antiplatelet drug resistance is an important issue in modern cardiovascular research [80]. Many studies have shown that PBCRBSCM may play a protective role in the treatment of antiplatelet drug resistance. The results of a randomized controlled trial involving 135 patients with stable angina pectoris in China showed that the combined use of *Salvia miltiorrhiza* polyphenolate injections and aspirin could significantly improve the sensitivity of thromboelastography, without the risk of bleeding [81]. A systematic review of 18 randomized controlled trials involving 1,460 patients with aspirin resistance showed that PBCRBSCM combined with aspirin could significantly reduce the platelet aggregation rate induced by ADP and AA in patients with aspirin resistance [82]. Similar systematic reviews have also reached similar conclusions and found that Tongxinluo capsules, Danshen preparations, leech extracts, and other PBCRBSCMs may play an important role in reducing aspirin resistance [83]. There are relatively few studies on the use of PBCRBSCMs to reduce clopidogrel resistance. Some studies believe that Danshen can inhibit cytochrome carboxylesterase and cytochrome P450 1A2, thereby affecting the metabolism of clopidogrel [84]. Another randomized controlled trial involving 49 clopidogrel resistant patients found that Xuefu Zhuyu decoction improved platelet function in patients resistant to clopidogrel, and its mechanism may be related to the inhibition of P2Y12 [85, 86].

In summary, PBCRBSCMs and their active ingredients can reduce the resistance to aspirin and clopidogrel, so that the combination of drugs can exert antiplatelet effects. However, the current research methods are heterogeneous, and the quality of research still needs to be improved, which further confirms the above conclusions.

## 5. The Efficacy of PBCRBSCM Combined with Antiplatelet Drugs in Ischemic Heart Disease

Several clinical studies have confirmed that PBCRBSCMs and their active ingredients combined with antiplatelet drugs and other conventional Western medicines have significant advantages in the treatment of coronary heart disease and angina. A meta-analysis of 14 randomized controlled trials including 1,367 patients with angina pectoris showed that compared with aspirin treatment alone, aspirin combined with compound Danshen dripping pills showed significant alleviation of angina pectoris symptoms and significantly improved the total clinical effective rate of patients with coronary heart disease [87]. Similar systematic reviews have confirmed that the combination of Tongmai Yangxin Pills [88], Kudiezi injections [89], *Salvia miltiorrhiza* polyphenolate injections [84, 90], and other PBCRBSCMs can improve the ECG findings of patients with angina pectoris and their clinical symptoms [91].

PBCRBSCM is often used as an adjuvant treatment method in the perioperative percutaneous coronary intervention (PCI) in patients with the acute coronary syndrome. Zhang et al. constructed a randomized controlled trial that included 136 patients with the acute coronary syndrome who underwent PCI. The patients were randomized to receive placebo or Tongxinluo capsule treatment in addition to the standard dual antiplatelet therapy of aspirin and clopidogrel. The results showed that both groups of patients with high platelet reactivity were significantly reduced. The reduction in the Tongxinluo capsule combined treatment group was more obvious than that in the aspirin and clopidogrel groups. Further studies have confirmed that its mechanism is related to the downregulation of P2Y12 response units and C-reactive protein levels [92]. A meta-analysis of 68 randomized controlled trials involving 6,043 patients showed that the combination of traditional Chinese medicine injection and conventional drugs, including aspirin and clopidogrel, is better than conventional drugs alone in terms of clinical efficacy and incidence of myocardial infarction [93].

In summary, PBCRBSCM combined with antiplatelet drugs and other conventional Western medicines confers therapeutic effects in the treatment of stable angina, unstable angina, and PCI during the perioperative period [94]. The effect of traditional Chinese medicine combined with antiplatelet drugs on the survival time of patients with ischemic heart disease remains to be confirmed by a large sample-sized, multicenter, randomized controlled study.

## 6. The Safety of PBCRBSCM Combined with Antiplatelet Drugs in Ischemic Heart Disease

Long-term use of antiplatelet drugs can lead to bleeding in patients with ischemic heart disease [95]. The dosage and duration of antiplatelet drugs should be strictly managed during antiplatelet therapy [96, 97]. Although the mechanisms of action of PBCRBSCM, when combined with antiplatelet drugs in the treatment of ischemic heart disease, have been studied in detail [98] and clinical studies have confirmed its effectiveness, the safety of PBCRBSCM remains worthy of attention.

Multiple clinical studies have explored the safety of the combination of PBCRBSCM and antiplatelet drugs. A randomized controlled trial involving 240 patients explored the efficacy and safety of Wufuxinnaoqing soft capsule in combination with antiplatelet drugs and other conventional drugs for the treatment of angina pectoris. The results confirmed that the incidence of adverse events in the combined treatment group was not significantly different from that in the Western medicine group [99]. Similar clinical trials have confirmed the safety of Shenzhu Guanxin Recipe [100]. A high-quality study evaluated the efficacy and safety of traditional Chinese medicine and its compounds in the treatment of atherosclerotic cardiovascular disease. The results suggested that there was no significant difference in the incidence of adverse events between various traditional Chinese medicines, including Radix *Salvia miltiorrhiza*, Rhizoma Ligustici Chuanxiong, Flos Carthami, and Tongxinluo capsule, Xinyue capsule, and Tongmaiyangxin pill, when compared with the Western medicine control group. [101]. Systematic reviews have confirmed the safety of *Panax notoginseng* saponins [102].

Overall, the safety of the combined use of PBCRBSCM and antiplatelet drugs has been supported by clinical trials [103]. Compared with the Western medicine group alone, combined Chinese medicines did not significantly increase or reduce the incidence of cardiovascular adverse events. However, there is a lack of systematic and long-term summary of the safety of the combination of PBCRBSCM and antiplatelet drugs [104]. The registration system for clinical adverse events may provide a new perspective for the safety evaluation of PBCRBSCM.

## 7. Concluding Remarks

PBCRBSCM is often used to treat ischemic heart disease [101, 105]. Studies have shown that PBCRBSCM can inhibit the adhesion, activation, and aggregation of platelets [106, 107]. It mainly inhibits platelet adhesion by downregulating vWF, interfering with collagen receptors, and protecting the vascular endothelium. Preventing platelet activation involves inhibiting the binding of ADP to P2Y1 and P2Y12 receptors on platelets and subsequently inhibiting the synthesis of PAF and TXA2. Inhibition of platelet aggregation is mainly related to the inhibition of the activation of integrin-*α* IIb/*β*3 and downregulation of FIB and vWF expression.

PBCRBSCM can be used in combination with antiplatelet drugs to exert antiplatelet effects [108, 109]. A large number of experimental studies have confirmed that the mechanism of action of some PBCRBSCMs and their active ingredients combined with conventional antiplatelet drugs is mainly related to the inhibition of platelet activation and aggregation, improvement of hemodynamic status and coagulation function, and correction of metabolism and inflammation. PBCRBSCMs can regulate the absorption and metabolism of conventional antiplatelet drugs and protect the vascular endothelium. Simultaneously, they regulate the inflammatory and AA/COX/PG pathways, exert a protective effect on gastric mucosal epithelial cells, inhibit the occurrence of ulcers, and reduce gastric mucosal damage induced by conventional antiplatelet drugs. In clinical studies of patients with ischemic heart disease, PBCRBSCMs and their active ingredients reduced the resistance to aspirin and clopidogrel, and when combined with conventional antiplatelet drugs, they exerted an antiplatelet effect.

A large number of randomized controlled trials and meta-analyses have confirmed that PBCRBSCM combined with antiplatelet drugs and other conventional Western medicines confers therapeutic effects in patients with stable and unstable angina, and the perioperative period in patients undergoing PCI. The safety of the combined use of PBCRBSCM and antiplatelet drugs has been supported by clinical trials. Compared with Western medicine alone, combined treatment with Chinese and Western medicine did not significantly increase or reduce the incidence of cardiovascular adverse events. Considerable progress has been made in the research on the antiplatelet mechanism of PBCRBSCM, but most clinical studies have limitations such as small sample sizes and unreasonable research designs. This limits the translational application of PBCRBSCM as antiplatelet agents in clinical settings. Therefore, to generate conclusive results, a large sample-sized, multicenter, randomized controlled study is needed on the combined application of PBCRBSCM and antiplatelet drugs, with cardiovascular events as the endpoint index. Such a study will provide high-level evidence for the use of PBCRBSCM as antiplatelet agents in the treatment of ischemic heart disease.

## Figures and Tables

**Figure 1:** PBCRBSCMs that are widely used in antiplatelet therapy. (a) Radix et rhizoma salviae miltiorrhizae, (b) rhizoma chuanxiong, (c) radix et rhizoma notoginseng, (d) radix paeoniae alba, and (e) flos carthami.

**Figure 2:** Active ingredients of PBCRBSCMs with antiplatelet effect. (a) Tanshinone IIA, (b) tetramethylpyrazine, (c) paeoniflorin, (d) salvianolic acid B, and (e) notoginsenoside Fc.

**Figure 3:** Pharmacological mechanism underlying the antiplatelet effect of PBCRBSCM. PBCRBSCM: Chinese medicine for promoting blood circulation and removing blood stasis; cAMP: cyclic adenosine monophosphate; cGMP: cyclic guanosine monophosphate; FIB: fibrinogen; vWF: von Willebrand factor; P2Y12: P2Y purinoceptor 12; PAC-1: procaspase activating compound-1; TXA2: thromboxane A2; PGI2: prostaglandin I2; ADP: adenosine diphosphate; PAF: platelet-activating factor; AA: arachidonic acid; Erk: extracellular signal-regulated kinase; SIRT1: silent mating type information regulation 2 homolog 1; NO: nitric oxide; Nrf2: nuclear factor erythroid 2-related factor 2; PI3K: phosphoinositide 3-kinase; MAPK: mitogen-activated protein kinase; NF-*κ*B: nuclear factor-kappa B.

**Figure 4:** The mechanism of the combined application of PBCRBSCM and antiplatelet drugs.
